# The association between sleep problems and general quality of life in cancer patients and in the general population

**DOI:** 10.3389/fpsyg.2022.960029

**Published:** 2022-12-15

**Authors:** Dirk Hofmeister, Thomas Schulte, Anja Mehnert-Theuerkauf, Kristina Geue, Markus Zenger, Peter Esser, Heide Götze, Andreas Hinz

**Affiliations:** ^1^Department of Medical Psychology and Medical Sociology, Leipzig University, Leipzig, Germany; ^2^Rehabilitation Clinic Bad Oexen, Bad Oeynhausen, Germany; ^3^Department of Applied Human Studies, University of Applied Sciences Magdeburg-Stendal, Stendal, Germany; ^4^Integrated Research and Treatment Center Adiposity Diseases, Leipzig University, Leipzig, Germany

**Keywords:** cancer, insomnia, sleep loss, quality of life, age differences, sex differences

## Abstract

**Objective:**

It is well-known that patients with cancer frequently experience sleep problems, and that sleep quality is associated with general quality of life (QoL). The aims of this study were to analyze the relationship between sleep problems and other components of QoL in more detail and to investigate sex and age differences in sleep quality in cancer patients in comparison with the general population.

**Method:**

This study comprised one general population sample (*n* = 4,476) and eight samples with cancer patients (*n* between 323 and 4,020). Sleep Quality was measured using the QoL questionnaire EORTC QLQ-C30.

**Results:**

All of the cancer patient groups reported more sleep problems than the general population. Sleep problems were associated with all facets of QoL both in cancer patients and in the general population. The highest associations were found in cancer patients for *fatigue* (*r* = 0.52) and *emotional functioning* (*r* = −0.47). The association between sleep quality and general QoL was lower in the cancer samples (*r* = −0.37) than in the general population (*r* = −0.46). Female cancer patients reported markedly more sleep problems than male patients did (*d* = 0.45), while this sex difference was lower in the general population (*d* = 0.15). In contrast to the general population, younger cancer patients had greater trouble sleeping than older patients did (*d* = −0.17).

**Conclusion:**

The results underline the significance of the role mental factors play in sleep problems. Health care providers should pay special attention to female patients and younger patients concerning this issue.

## Introduction

According to the WHO, the number of cancer-related deaths is about 10 million worldwide, and the number is expected to increase markedly in the next decades (Sung et al., 2021).

Cancer patients often experience sleep disturbances (Ancoli-Israel, 2009; Akman et al., 2015; Otte et al., 2015; Strik et al., 2021), the prevalence of which ranges from 30 to 93% (Lin et al., 2020). Sleep problems often remain undetected in clinical practice (Kwak et al., 2020), and they are common among cancer survivors even after cancer treatment completion (Schieber et al., 2019; Aronsen et al., 2022). They are associated with reduced quality of life (QoL; Ancoli-Israel et al., 2014), depression (Hofmeister et al., 2020), concentration problems (Henneghan et al., 2018), fatigue (Medysky et al., 2017; Chartogne et al., 2021), and even reduced survival (Gottfried et al., 2020; Bach et al., 2021). However, it has yet to be systematically examined whether sleep problems are more strongly associated with physical health or with mental health problems, and previous studies have had inconsistent findings. While some found no difference between physical health and mental health in terms of how those dimensions were correlated with sleep problems (Kudielka et al., 2004), some detected stronger associations between sleep problems and physical health problems (Delgado-Guay et al., 2011; Sandadi et al., 2011), and others reported stronger associations with mental health factors (Nock et al., 2020; Pozzar et al., 2021).

Sex and age differences in sleep quality have been examined in both patient and general population samples. Most studies have found that females report having greater trouble sleeping than males do, while no consistent age effects were observed (Hinz et al., 2017a; Tibubos et al., 2020; Santoso et al., 2021; Schulte et al., 2021). Since cancer types and sex as well as age can be confounded, it is important to quantify sex and age differences when the impact of specific cancer types or treatments on sleep quality is to be examined. Therefore, it is relevant to investigate sex and age effects on sleep quality in cancer patients, and, for reasons of comparability, in the general population as well. A further issue is the question whether the strengths of the associations between sleep quality and general QoL depend on sex and age, e.g., whether sleep quality predicts QoL better or worse in samples of females in comparison with samples of males. This issue has not been addressed previously.

The relationship between sleep quality and other aspects of QoL, as well as age and sex effects, have been investigated in many studies that used a variety of questionnaires and many different samples of cancer patients. This makes it difficult to generalize the results. In our study, we used a single questionnaire, the EORTC QLQ-C30, which measures multiple components of QoL, including sleep quality, in a uniform way. Eight sufficiently large samples of cancer patients were included, making it possible to cover a wide range of cancers and settings. The results of the cancer samples are contrasted with a large sample of individuals from the general population to show the extent to which the associations of the QoL components and the age and sex effects found in the cancer samples are also present in the general population.

Summing up, the aims of this study were (a) to analyze the associations between sleep quality and other aspects of QoL in cancer patients, and to compare these results with the associations found in the general population, (b) to investigate sex and age effects on sleep quality in both types of samples, and (c) to explore sex and age effects of the correlations between sleep quality and general QoL assessments.

## Methods

This study is a summarizing analysis of results obtained from several samples. The data set consists of eight German samples of cancer patients and one German general population sample. These samples have already been analyzed and featured in published studies with other objectives. Table 1 shortly describes the samples and references where further aspects of the studies such as sampling procedure, sociodemographic and clinical characteristics, time of examination, and response rate are described. The analyses were restricted to the respondents for whom sleep scale scores were available. Therefore, the sample sizes are not always exactly identical to those described in the reference papers. All of the studies were approved by corresponding ethics committees, and informed consent was obtained from all participants.

**Table 1:** Characteristics of the samples.

	General population	MIXED	REHA I	REHA II	URO-GYN	GYN	BREAST	HEMA	AYA
*n*	4,476	4,020	1,225	2,059	433	354	323	1,288	514
Age (years) M	50.1	58.4	55.8	62.4	60.7	61.2	66.2	61.0	30.1
(SD)	(17.1)	(11.3)	(16.0)	(14.2)	(10.5)	(14.2)	(9.6)	(14.9)	(6.2)
Range	18–92	18–92	18–88	18–92	19–81	23–88	31–85	19–86	18–41
Sex (% Females)	54.7	51.4	52.2	41.2	25.4	100	100	45.4	75.1
References	Hinz et al. (2014)	Mehnert et al. (2014)	Friedrich et al. (2019)	Hinz et al. (2015)	Zenger et al. (2010, 2011)	Thieme et al. (2017)	Fuhrmann et al. (2015)	Esser et al. (2018)	Leuteritz et al. (2018)

In all eight clinical samples, general inclusion criteria were a confirmed cancer diagnosis, age 18 years or older, and sufficient cognitive ability and language skills to complete the questionnaires. In samples 2 through 7, patients were visited in person and asked to participate; in samples 8 and 9, both personal visit and request to participate in an online survey were used. Samples 7 and 8 had completed treatments; the remaining clinical samples included patients with both completed and non-completed treatments. Samples 1, 2, 4, and 8 were cross-sectional studies; the remaining samples were longitudinal studies, but for these studies only the first measurement time point is considered here.

### Sample 1: General population

This sample was compiled from two surveys conducted in Germany. In both surveys, the samples were fairly representative of the German population living in private homes in terms of age and sex distribution. Both samples are described in more detail elsewhere (Hinz et al., 2014). The sample sizes were *n* = 2,448 for subsample 1 and *n* = 2,028 for subsample 2, resulting in a total sample of *n* = 4,476.

### Sample 2: MIXED – Mixed cancer patients

This multicenter study included 4,020 cancer patients receiving treatment in acute care hospitals, outpatient facilities, and rehabilitation clinics. The most frequent cancer localizations were: breast (22%), digestive organs (20%), and male genital organs (17%). Five study centers in Germany were involved in this project (Mehnert et al., 2014).

### Sample 3: REHA I – Mixed cancer patients in rehabilitation clinic I

Sample 3 was composed of cancer patients enrolled in a rehabilitation program to regain physical fitness (*n* = 1,225). The most frequent cancer diagnoses were breast cancer (25%), prostate cancer (19%), and cancer of the gastrointestinal tract (18%; Friedrich et al., 2019).

### Sample 4: REHA II – Mixed cancer patients in rehabilitation clinic II

Sample 4 also included cancer patients participating in a rehabilitation program (*n* = 2,059). The tumor sites with the highest frequency were prostate (31%), breast (17%), colon (9%), and kidney (6%). The participants of this study were sent the questionnaire 6 months after finishing the rehabilitation program (Hinz et al., 2015).

### Sample 5: URO-GYN – Urological and gynecological cancer patients

Sample 5 was composed of 323 male patients with urologic cancer (Zenger et al., 2010) and 110 female patients with gynecological cancer (Zenger et al., 2011) receiving treatment in a university hospital. In this analysis, we only use the data from the first measurement point (t1), obtained in hospital.

### Sample 6: GYN – Gynecologic cancer patients

Patients with gynecological or breast cancer (*n* = 354) were consecutively recruited for this study in the gynecological clinics of three German hospitals. As in Sample 5, we only use the data from the first measurement point obtained in hospital (Thieme et al., 2017).

### Sample 7: BREAST – Breast cancer patients

Sample 7 consists of 323 women who took part in a routine radiologic after-treatment (breast cancer) examination. Directly after the radiologic examination, the participants were asked to complete the questionnaires (Fuhrmann et al., 2015).

### Sample 8: HEMA – Hematological cancer survivors

This sample included survivors of hematological malignancies (≥2.5 years after diagnosis) from two German cancer registries (Esser et al., 2017). The most frequent cancer types were non-follicular lymphoma (27%), lymphoid leukemia (15%), and follicular lymphoma (13%). While the publication describing the study methods (Esser et al., 2018) included only 922 patients, our sample was enlarged with further hematological survivors and reached a sample size of *n* = 1,288.

### Sample 9: AYA – Adolescents and young adults

A sample of 514 AYAs (age 15–39 years at diagnosis) was included in this study. The most common tumor diagnoses were breast (27%), non-Hodgkin lymphoma (18%), gynecological tumors (9%), testicular tumor (8%), and hematological cancer (7%). Patients were recruited in 16 German acute care hospitals, four rehabilitation centers, and from two cancer registries (Leuteritz et al., 2018).

### Instrument

The 30 items of the EORTC QLQ-C30 (Aaronson et al., 1993) are distributed across five functioning scales, 9 symptom scales (including single symptom items and an item reflecting financial difficulties), and a 2-item global health/QoL scale. Items 1–28 have four possible response options (not at all, a little, quite a bit, very much), and the remaining two items have seven. High functioning scales, global health/QoL scale, and sum scores represent high QoL, while high scores on the symptom scales (including sleep problems) indicate low QoL. The EORTC Quality of Life Group proposed a summarizing score of higher order (sum score) which is composed of the five functioning scales and eight symptom scales (Giesinger et al., 2016).

In our analyses, we focused on the one-item sleep scale of the EORTC QLQ-C30:

“(During the past week): Have you had trouble sleeping?,” with the four response categories from “not at all” to “very much.” The raw scores are transformed linearly to a scale from 0 to 100, where a high score represents more sleep problems. The validity of this scale was underlined by the correlation between this one-item scale and the Jenkins Sleep Scale of 0.73 (Hofmeister et al., 2020) in a large sample of mixed cancer patients and between 0.74 and 0.81 in colorectal cancer survivors (Legg et al., 2022). Moreover, the association between the EORTC QLQ-C30 sleep scale and the 18-item Karolinska Sleep Questionnaire was characterized by an odds ratio of 8.2 (Lagergren et al., 2021) in a study with esophageal cancer patients. Normative values of the EORTC QLQ-C30 including the sleep scale are available for several countries (Hinz et al., 2014; Nolte et al., 2019).

### Statistical analysis

Associations between the sleep scale and other scales are expressed with Pearson correlation coefficients. Pearson correlations were used because they provide the best comparability with results from the literature. For characterizing group differences, we used effect sizes *d*, relating the mean score differences of the groups to the pooled standard deviations. The two age groups were defined as ≤59 years vs. ≥ 60 years for all of the samples except the AYA. Because of the non-normality of the distribution of correlation coefficients, the mean correlations across the eight cancer samples were calculated *via* Fisher’s z-transformation of the single coefficients. For this averaging procedure, we gave each sample the same weight and did not use weighting factors according to the sample sizes because we intended to represent each setting underlying the samples with the same weight. All calculations were performed with SPSS version 27.

## Results

### Correlations between sleep problems and other scales

Table 2 presents the correlations between the sleep scale and the other scales of the EORTC QLQ-C30. Sleep quality was significantly correlated with all components of QoL in all of the samples; positive correlations were found with the symptom scales, and negative correlations with the functioning scales, the global QoL scale, and the sum score. In both types of samples, the general population and the cancer patients, the strongest associations were found for fatigue and for emotional functioning. The correlations in the general population sample were generally stronger than those in the cancer patient samples.

**Table 2:** Correlations between the sleep scale and the other scales.

	General population	MIXED	REHA I	REHA II	URO-GYN	GYN	BREAST	HEMA	AYA	CA-Mean
	*n* = 4,476	*n* = 4,020	*n* = 1,225	*n* = 2,059	*n* = 433	*n* = 354	*n* = 323	*n* = 1,288	*n* = 514
Physical functioning	−0.43	−0.33	−0.33	−0.37	−0.41	−0.24	−0.22	−0.37	−0.32	−0.33
Role functioning	−0.41	−0.32	−0.35	−0.38	−0.53	−0.42	−0.28	−0.42	−0.36	−0.38
Emotional functioning	−0.50	−0.45	−0.46	−0.49	−0.50	−0.42	−0.44	−0.52	−0.45	−0.47
Cognitive functioning	−0.47	−0.36	−0.38	−0.33	−0.51	−0.40	−0.27	−0.44	−0.41	−0.39
Social functioning	−0.43	−0.30	−0.33	−0.35	−0.42	−0.45	−0.27	−0.41	−0.30	−0.36
**Global health /QoL**	**−0.46**	**−0.38**	**−0.33**	**−0.39**	**−0.48**	**−0.30**	**−0.26**	**−0.40**	**−0.41**	**−0.37**
Fatigue	0.60	0.46	0.49	0.51	0.65	0.52	0.43	0.56	0.53	0.52
Nausea/ vomiting	0.30	0.18	0.21	0.19	0.40	0.27	0.15	0.28	0.18	0.23
Pain	0.47	0.36	0.41	0.38	0.55	0.45	0.32	0.42	0.35	0.41
Dyspnea	0.38	0.24	0.26	0.30	0.35	0.33	0.31	0.33	0.31	0.30
Insomnia	1	1	1	1	1	1	1	1	1	1
Appetite loss	0.40	0.26	0.27	0.29	0.54	0.45	0.27	0.35	0.32	0.35
Constipation	0.25	0.20	0.18	0.23	0.38	0.19	0.12	0.25	0.23	0.22
Diarrhea	0.20	0.16	0.13	0.20	0.30	0.09	0.20	0.20	0.23	0.19
Financial difficulties	0.34	0.18	0.20	0.28	0.21	0.27	0.19	0.29	0.22	0.23
**Sum score**	**−0.70**	**−0.58**	**−0.61**	**−0.56**	**−0.74**	**−0.65**	**−0.54**	**−0.64**	**−0.64**	**−0.62**

CA-Mean, Mean score of the eight cancer samples. Bold, correlations with the Global health/QoL scale and with the sum score.

### Sex and age differences in sleep problems

Regarding the overall comparison between the clinical samples and the general population, the bottom rows of Table 3 show that sleep problems were markedly more frequent in all clinical samples (*M* between 32.6 and 54.7) than in the general population (*M* = 14.3).

**Table 3:** Mean scores of the sleep scale, broken down by sex and age group.

	General population	MIXED	REHA I	REHA II	URO-GYN	GYN	BREAST	HEMA	AYA	CA-Mean
**Sex**										
Males M	12.2	37.9	47.1	26.8	26.9	–	–	29.5	27.8	32.7
(SD)	(23.6)	(36.4)	(35.0)	(30.8)	(33.1)	–	–	(32.0)	(31.4)	(33.1)
Females M	15.9	48.0	61.6	43.9	49.1	–	–	43.4	44.0	48.3
(SD)	(26.4)	(37.7)	(35.2)	(35.0)	(38.8)	–	–	(36.3)	(37.1)	(36.6)
Effect size	0.15	0.27	0.41	0.52	0.62	–	–	0.41	0.47	0.45
**Age group**										
≤59 years M	10.3	46.4	56.9	36.0	38.5	46.8	46.8	40.1	–	44.5
(SD)	(22.1)	(37.6)	(35.8)	(33.5)	(38.1)	(37.0)	(33.9)	(36.3)	–	(36.0)
≥60 years M	22.2	40.0	52.1	32.8	28.8	40.2	41.8	32.8	–	38.4
(SD)	(29.1)	(37.0)	(35.8)	(33.7)	(34.0)	(34.7)	(34.7)	(33.0)	–	(34.7)
Effect size	0.46	−0.17	−0.13	−0.10	−0.27	−0.18	−0.15	−0.21	–	−0.17
**Total sample**										
M	14.3	43.1	54.7	33.8	32.6	42.9	42.9	35.8	40.0	40.7
(SD)	(25.3)	(37.4)	(35.9)	(33.6)	(35.9)	(35.8)	(34.6)	(34.7)	(36.4)	(35.5)

CA-Mean, Mean score of the eight cancer samples; M, Mean; SD, standard deviation.

Females reported more sleep problems than males in all samples (Table 3), and the effect sizes of this sex difference were higher in the clinical samples (*d* between 0.27 and 0.62) than in the general population (*d* = 0.15). Younger patients reported more sleep problems than older patients in all of the clinical samples, while the opposite was true of the general population sample. The GYN and BREAST samples included only women, and the AYA sample was composed entirely of young patients; therefore, the corresponding group differences could not be calculated in Table 3.

### Relationship between sleep quality and global QoL

Table 4 presents the correlations between the sleep scale and the two-item global health/QoL scale, separately for males and females and for younger and older patients. All coefficients are negative, thus indicating decreasing QoL with increasing sleep problems. Correlations across the total samples are presented above in Table 2. In most of the samples, the correlations were slightly higher in the subsample of males compared those in the women’s groups, and the correlations among the younger patients were generally somewhat stronger than those among the older patients.

**Table 4:** Correlations between the sleep scale and global QoL, broken down by sex and age group.

	General population	MIXED	REHA I	REHA II	URO-GYN	GYN	BREAST	HEMA	AYA	CA-Mean
**Sex**										
Males	−0.48	−0.44	−0.39	−0.43	−0.46	–	–	−0.39	−0.43	−0.42
Females	−0.45	−0.33	−0.36	−0.33	−0.36	–	–	−0.41	−0.39	−0.36
**Age group**										
≤59 years	−0.44	−0.36	−0.41	−0.40	−0.58	−0.50	−0.40	−0.47	–	−0.45
≥60 years	−0.41	−0.40	−0.35	−0.38	−0.39	−0.15	−0.22	−0.35	–	−0.32

CA-Mean, Mean of the eight cancer samples.

## Discussion

All cancer groups reported markedly higher levels of sleep problems than the general population. This finding is not new, and confirms results often reported in the literature. The first specific research question of the present study concerned analyzing the association between sleep quality and QoL. Sleep quality was significantly correlated with all components of QoL in all samples. In both types of sample groups, the general population and the cancer patients, the highest associations were found for *fatigue* and *emotional functioning*, while the lowest associations were observed for the specific symptoms *diarrhea*, *constipation*, *nausea*/*vomiting*, and *financial difficulties*. It is interesting to note that the psychological QoL dimensions, *emotional* and *cognitive functioning*, are more strongly correlated with sleep problems than are the more physical components, *physical functioning* and *role functioning*. The term fatigue comprises physical as well as mental components, and fatigue proved to be the scale with the highest associations with sleep problems of all of the nine samples. In a study on disruptive factors that may explain why cancer patients experience the sleep problems they do, psychological factors such as *worrying* had a stronger prognostic power than objective and physical factors such as *nocturnal urination* or *pain* (Schulte et al., 2021) did, a finding that further underlines the relevance of mental factors in the prognosis of sleep problems.

A further result was that all correlations between sleep quality and QoL in the general population group were higher than the mean correlations of the cancer patients. While the correlations between sleep problems and the 2-item general health/QoL scale was *r* = −0.46 in the general population sample, the mean correlation of the cancer samples was only *r* = −0.37. This indicates that sleep problems are more relevant for the prediction of general QoL in the general population as compared with cancer patient groups. At first glance, this seems to contradict the importance of sleep problems among cancer patients. In our study, the magnitude of sleep problems was markedly higher in all cancer patient samples than in the general population. However, the lower correlations in the cancer groups actually mean that the sleep disturbances are not as strongly associated with other detriments to QoL as they are in the general population, and that they cannot be predicted very well by the other variables. In contrast to cancer patients, sleep problems experienced by members of the general population may be the only problem that person has, and thus explains why a stronger association between sleep quality and general QoL exists in that general population group. Cancer patients, on the other hand, are faced with multiple other detriments in addition to having trouble sleeping. While this fact might reduce the relative importance of sleep quality for the general QoL assessment, it does not reduce the relevance of sleep problems *per se*.

The highest correlations found in Table 2 are those between sleep problems and the EORTC QLQ-C30 sum score. Here it must be taken into account however that the sleep problems are already included in the sum scores, and thus lead to a slight artificial inflation of the association. Nevertheless, a comparison between the different samples is possible, and, once more, the correlation is highest in the general population.

A further aim of the study was to investigate sex and age differences in sleep problems and their associations with QoL. It is well-known that females in general population samples report higher levels of sleep problems than males do (Hinz et al., 2017a). In our study, the relevant effect size was *d* = 0.15, a finding that is in line with other normative studies that have also used the EORTC QLQ-C30 for measuring sleep quality. Effect sizes with coefficients of *d* = 0.24 (Waldmann et al., 2013) and *d* = 0.13 (Nolte et al., 2020) can be inferred from two further German normative studies, and a large international normative study reported an effect size of *d* = 0.19 (Nolte et al., 2019). Females in our cancer samples also reported more sleep problems than males did. All eight samples showed more pronounced sex differences (mean effect size: *d* = 0.45) than the general population sample (*d* = 0.15), indicating that heightened sleep disturbances in female cancer patients are not only due to their sex. The threat of a cancer diagnosis provokes more sleep problems in female cancer patients in addition to their generally poorer sleep quality, a phenomenon which may be related to higher levels of anxiety (Hinz et al., 2017b) and fear of progression (Hinz et al., 2015) in females in comparison with males.

Regarding age, the cancer patient samples reported the opposite effect of that seen in the general population sample. In the latter, older people were more prone to sleep problems than younger ones, a fact that can also be observed in other normative studies (Hinz et al., 2014), while the younger cancer patients reported more sleep problems than the older ones. This confirms that a cancer diagnosis is particularly threatening for younger patients. Other studies have also found that, compared with their healthy peers, young cancer patients are more anxious and more depressed than older patients in relation to their healthy peers (Hinz et al., 2019).

As already mentioned above, our study confirmed severe sleep problems in cancer patients and clear associations between sleep quality and general QoL. While the QoL questionnaire EORTC QLQ-C30 has an item that measures sleep quality, the SF-36 does not. Unfortunately, most instruments for measuring supportive care needs such as the SCNS-SF34 (Boyes et al., 2009) or the CaSUN (Hodgkinson et al., 2007) do not cover sleep problems at all; therefore, these unmet needs may remain undetected. Many cancer patients find it easier to admit that they are having trouble sleeping than that they are experiencing depressive symptoms. Thus, talking about sleep problems can also serve as a path for facilitating support services for regaining mental health.

The take-away of this study for health care providers is that females and younger cancer patients deserve special attention concerning their sleep quality. This message is not new, but the compilation of the studies with different cancer types and different settings confirms the generalizability of this finding. Since sleep problems can become chronic when left untreated, health care providers should consider offering their patients who suffer from sleep problems intervention techniques for improving sleep quality such as physical exercise (Yang et al., 2021), behavioral or cognitive-behavioral treatment (Zhou et al., 2020; Savard et al., 2022), or stress reduction (Suh et al., 2021).

Some limitations of this study should be mentioned. The mean scores of the sleep scale for samples 2 and 4 have already been reported in previous publications (Hinz et al., 2017c; 2018), and for some of the samples mean scores of certain subsamples (but not the whole sample) have also been reported previously. However, the results on age and sex differences as well as the correlations between sleep problems and QoL, presented separately divided by sex and age, are new. The participants of the general population sample were on average somewhat younger than the cancer patients; therefore, some of the differences between the patients and the general population might, at least in part, be due to those mean age differences. The eight cancer samples were heterogeneous concerning multiple criteria such as tumor types, time since diagnosis, recruitment procedure, and other factors. Therefore, it is not possible to attribute differences between the eight cancer samples to just one cause. However, the heterogeneity of the cancer samples can also be seen as an advantage, as it allows for estimating the degree of generalizability of the results. The one-item sleep scale of the EORTC QLQ-C30 is less reliable than sleep scales with more items. However, the difference in accuracy between this single-item scale and more comprehensive scales is not severe (Hofmeister et al., 2020; Schulte et al., 2021), and the large sample sizes can compensate for inaccuracies in the sleep scale of the EORTC QLQ-C30 to a certain degree. In our analyses, we could not consider the influence of comorbidity (e.g., Ferro et al., 2020) and of medication (e.g., Voiss et al., 2019) on the relationship between sleep quality and QoL because the corresponding data on comorbidities and medication were not available.

Taken together, the present study contributes to clarifying the magnitude and role of sleep problems in the context of QoL. It underlines that sleep problems are severe in cancer patients, and it gives oncologists and other health care providers information concerning groups with specific needs, especially females and young cancer patients.

## Data availability statement

The data analyzed in this study is subject to the following licenses/restrictions: The datasets presented in this article are not readily available due to the heterogeneity of their origins. Requests for access to the datasets should be addressed to the corresponding authors of the original studies (Zenger et al., 2010, 2011; Hinz et al., 2014, 2015; Mehnert et al., 2014; Fuhrmann et al., 2015; Thieme et al., 2017; Leuteritz et al., 2018; Friedrich et al., 2019). Requests to access these datasets should be directed to andreas.hinz@medizin.uni-leipzig.de.

## Ethics statement

The studies involving human participants were reviewed and approved by the Ethical Review Board Leipzig University. The patients/participants provided their written informed consent to participate in this study.

## Author contributions

AH and DH designed the study, performed the statistical analyses, wrote the first draft, and wrote the final version. TS, AM-T, KG, MZ, PE, and HG recruited patients. AH obtained data from the general population. All authors contributed to the article and approved the final version.

## Funding

The original research was funded and supported by German Cancer Aid (Grant Numbers: 70112267, 107 447, 107465, and 110948) and German Research Foundation (Grant Number HI 1108/5-1). The authors acknowledge the support by the Open Access Publishing Fund of Leipzig University, supported by the German Research Foundation within the program Open Access Publication Funding.

## Conflict of interest

The authors declare that the research was conducted in the absence of any commercial or financial relationships that could be construed as a potential conflict of interest.

## Publisher’s note

All claims expressed in this article are solely those of the authors and do not necessarily represent those of their affiliated organizations, or those of the publisher, the editors and the reviewers. Any product that may be evaluated in this article, or claim that may be made by its manufacturer, is not guaranteed or endorsed by the publisher.
